This article has been retracted.

# Study on the Application and Efficacy of Responsibility Nursing in Dialysis Care

**DOI:** 10.1155/2021/2210191

**Published:** 2021-07-29

**Authors:** Ting Wu, Meiling Gao, Jun Shi, Linfang Xu, Jing Wang, Kaili Zhang

**Affiliations:** Blood Purification Center, Yanghu Branch of Changzhou Second People's Hospital, Changzhou 213000, Jiangsu, China

## Abstract

Providing high-quality care to patients undergoing hemodialysis (HD) is a priority for nurses. The present study was conducted to explore the experiences of the quality of nursing care among patients, nurses, and caregivers in Yanghu Branch of Changzhou Second People's Hospital, China. A total of 120 hemodialysis patients consecutively admitted to Yanghu Branch of Changzhou Second People's Hospital were enrolled and divided into two groups according to the nursing method they received: control group (routine nursing) and experimental group (responsibility nursing). The two cohorts were observed and compared for alterations of adverse emotions and inflammatory factors, the incidence of complications, pre-and post-nursing sleep quality, life quality, and patients' satisfaction with nursing. After nursing, the Self-Rating Anxiety/Depression Scale (SAS/DS) scores were lower in the experimental group (EG) than in the control group (CG) (both *P* < 0.05). Serum IL-6, hs-CRP, and TNF-*α* were decreased in both groups after nursing and were even lower in EG (both *P* < 0.05). EG had significantly improved sleep quality and life quality than CG, with a higher nursing satisfaction (all *P* < 0.05). This validates that the responsibility nursing for dialysis patients can validly mitigate patients' negative emotions, improve their quality of life, and ensure high-quality dialysis effect, which is feasible for wide popularization and application in clinics.

## 1. Introduction

Hemodialysis is the mainstay of treatment for end-stage renal disease (ESRD), defined as the final stage of the irreversible decline of renal function caused by various kidney diseases. At this stage, patients can only rely on renal replacement therapy to survive [1, 2]. There are currently three renal replacement therapy types for ESRD: hemodialysis, peritoneal dialysis, and kidney transplantation [3–5]. Of these, patients receiving hemodialysis occupy about 90% of the total number of dialysis patients [6]. The main contributing factors of ESRD include chronic glomerulonephritis [7], hypertensive kidney damage [8], diabetic nephropathy [9], rheumatic kidney damage [10], and polycystic kidney [11], among which chronic glomerulonephritis is the leading chronic kidney disease worldwide and also the main cause of ESRD [12]. Furthermore, recent years have witnessed an increasing proportion of ESRD caused by diabetes, as the number of diabetic patients increases with the continuous improvement of living standards and changes in lifestyle and diet [13]. Asymptomatic in the early stage, many patients with chronic kidney disease have entered the middle and late stages when they seek medical treatment. The symptoms appear clinically, increasing the treatment difficulty and bringing heavy economic and psychological burden to patients.

Moreover, the treatment of patients undergoing long-term dialysis is often complicated with cardiovascular and cerebrovascular diseases, anemia, renal osteopathic medicine, metabolic acidosis, electrolyte disorder, and other complications [14, 15]. Furthermore, they are susceptible to dialysis-related depression, a type of somatic depression referring to a group of diseases with depressive symptoms caused by long-term maintenance hemodialysis (MHD) [16]. Epidemiological investigation shows that the prevalence rate of depression in maintenance hemodialysis patients is 22.8%–62.0% [17]. Depression will affect patients' treatment compliance and quality of life, which will reduce their survival hope, increase the possibility of developing negative and even desperate thoughts, and even contribute to the decision to terminate dialysis. Apart from that, the mental stress and life burden brought by long-term dialysis are inevitable.

Therefore, it is essential to implement correct and effective nursing measures in long-term dialysis. The nursing staff's technical level and nursing quality will significantly affect the quality of dialysis and the quality of life of patients [18]. The responsibility nursing model is a kind of patient-centered model, providing comprehensive, systematic, and holistic nursing for patients' physical and mental health [19]. As one of the new nursing models, it can effectively ensure the provision of high-quality nursing care for patients. Accordingly, this study mainly focuses on the application and effect of responsibility nursing in dialysis nursing and has obtained satisfactory results, specifically, as follows.

The rest of the paper is structured as follows.  Section 2 describes material and methods. Then, in Section 3, results are discussed.  Section 4 is about discussion, and finally, the conclusion is presented in Section 5.

## 2. Materials and Methods

### 2.1. Research Participants

This study enrolled 120 hemodialysis patients treated in Yanghu Branch of Changzhou Second People's Hospital from September 2015 to September 2020 and divided them into control group (CG) and experimental group (EG) according to different nursing schemes. Patient clinical data were also collected. There were 54 patients in CG, including 29 males and 25 females, with an average age of (41.92 ± 5.67) years and an average dialysis time of (3.43 ± 0.84) years. EG (*n* = 66) consisted of 38 males and 28 females, with an average age of (43.24 ± 6.04) years and an average dialysis time of (3.58 ± 0.97) years. The general data were similar in both groups, as shown in Table 1 (*P* < 0.05, Table 1), indicating the comparability for further research. All patients were conscious and able to complete the questionnaire independently. Patients with severe complications, dysfunction of vital organs such as heart and liver, and cognitive impairment were excluded. An informed consent form was also obtained before enrollment.

### 2.2. Nursing Plan

Patients in CG received routine nursing, including instructing patients to follow the doctor's advice, appropriate health education, and in-patient nursing measures. Patients in EG were treated with responsibility nursing. After the implementation of responsibility nursing, every patient can get better recuperation.

They provided at least 2-3 shift nurses and a regular dialysis machine. The specific measures included dialyzer preflushing, patient condition evaluation, and establishment of cardiopulmonary bypass and measurement of patient's vital signs during dialysis treatment, machine monitoring, and drug use during and after dialysis. In addition, the nursing staff informed patients of the way, process, necessity, and significance of hemodialysis, to gain patients' trust and make them actively cooperate during hemodialysis treatment. After treatment, the dialysis unit was disinfected, and the patient's condition and machine operation status were recorded in time. Furthermore, patients were instructed to have a reasonable diet. The communication between nurses and patients was also strengthened. Moreover, psychological counseling was carried out to improve the psychological state of patients, eliminate negative emotions, and ensure the treatment effect.

### 2.3. Endpoints

Self-rating anxiety/depression scales (SAS/SDS) were used to evaluate the emotional changes of patients before and after nursing. The higher the score, the more serious the anxiety and depression.

Alterations of inflammatory factors including interleukin-6 (IL-6), high-sensitivity C-reactive protein (hs-CRP), and tumor necrosis factor *α* (TNF-*α*) were also compared. The lower the inflammatory factor level, the better the nursing effect. The Pittsburgh Sleep Quality Index (PSQI) was used for evaluation, including subjective sleep quality, sleep latency, sleep duration, habitual sleep efficiency, sleep disturbances, and use of sleeping medication, with a score ranging from 0 to 3 for each item. The higher the score, the more acute the sleep disturbance. The Generic Quality of Life Inventory-74 (GQOL-74) was employed to evaluate patients' quality of life before and after nursing from the dimensions of physical functioning, psychological functioning, social functioning, and material life. The higher the score, the higher the quality of life. The complications that occurred during treatment were observed and counted.

Nursing satisfaction was evaluated by the self-made nursing satisfaction questionnaire in our hospital, which was scored from five aspects: environmental satisfaction, service attitude satisfaction, technical satisfaction, life care satisfaction, and health education satisfaction.

### 2.4. Statistical Processing

SPSS 21.0 statistical software was used to analyze the research data. The mean and standard deviation (mean ± standard) of the data was measured. They were compared by t-test and chi-square test, respectively, with *P* < 0.05, indicating significant differences.

## 3. Results

### 3.1. Adverse Emotion Scores in Two Groups

SAS and SDS results revealed that both groups of patients had anxiety and depression before nursing with no significant differences between the two cohorts (*P* < 0.05). However, after nursing, SAS and SDS scores decreased in both groups and were even lower in EG (*P* < 0.05).  Table 2 shows that, after nursing, the SAS scores in CG and EG were 42.48 ± 3.14 and 36.14 ± 2.87, respectively, which are lower than the SAS scores before nursing, i.e., 56.51 ± 3.58 and 56.77 ± 3.71. Likewise, the SDS scores in both the groups after nursing were 40.58 ± 3.69 and 34.19 ± 2.97, which are significantly lower than the SDS scores before nursing. This shows that nursing has significantly reduced the anxiety and depression levels in both groups.

### 3.2. Levels of Inflammatory Factors in Two Groups

Figure 1 shows the results for serum inflammatory factors in both groups. Serum inflammatory factors were measured before and after nursing. IL-6, hs-CRP, and TNF-*α* were insignificantly different between CG and EG before nursing (*P* < 0.05). All the factors were reduced after nursing, with lower parameters in EG (*P* < 0.05).

### 3.3. Comparison of Sleep Quality between Two Groups

Table 3 shows the results for subjective sleep quality, sleep latency, sleep duration, habitual sleep efficiency, sleep efficiency, and use of sleep medication in both the control and experimental group. It is evident that, after nursing, the scores for all these measures were significantly reduced. For example, before nursing, the subjective sleep quality and sleep latency in CG were 2.45 ± 0.19 and 2.67 ± 0.26, respectively. After nursing, these scores were reduced to 1.52 ± 0.09 and 1.73 ± 0.18.

### 3.4. Comparison of Life Quality between Two Groups

Before and after nursing, the quality of life of patients was evaluated by GQOL-74 from the four dimensions of physical functioning, material life, psychological functioning, and social functioning. The scores for all dimensions were similar in the two groups before nursing (*P* < 0.05) but were higher in EG than in CG post-nursing (*P* < 0.05).  Table 4 shows the results for quality of life scores in both groups. For example, before nursing, the physical functioning score for both the groups were 58.86 ± 4.25 and 59.24 ± 4.77, respectively, which are lower than physical functioning score after nursing, i.e., 60.48 ± 3.87 and 68.74 ± 3.54.

### 3.5. Incidence of Complications in Two Groups

Complications of hemodialysis mainly include dialysis membrane rupture, mild coagulation, and hypotension during dialysis. The incidence of complications in EG was 7.5%, a rate lower than 20.3% in CG (*P* < 0.05).  Table 5 provides the details for the incidence of complication in both groups.

### 3.6. Nursing Satisfaction of Patients in Two Groups

The self-made nursing satisfaction questionnaire was used to evaluate patients' nursing satisfaction.  Table 6 provides the scores for satisfaction levels in both EG and CG groups. The results demonstrated that patients' satisfaction in EG was higher than that in CG in terms of environment, service attitude, technical level, life care, and health education (*P* < 0.05).

## 4. Discussion

Hemodialysis is to draw the patient's blood out of the body and remove some harmful substances through certain devices and purify the blood, called blood purification [20]. The primary purpose of hemodialysis is to remove excessive toxic substances and water retained in the patient's body while supplementing the substances needed in the body to maintain the relative stability of the patient's internal environment. So, instead of completely replacing the original function of the kidney, hemodialysis can only partially replace a certain part of the function of the kidney [21]. Blood purification treatment is a highly technical nursing task in which nurses play a significant role, with higher requirements for their sense of responsibility. The implementation of responsibility nursing can fully guarantee the quality of nursing service for patients [22]. In the process of dialysis, the nursing staff can effectively improve patients' nursing satisfaction and finally obtain significant nursing effect by giving patients dietary guidance and explaining the related knowledge of diseases.

This study compared the curative effect of hemodialysis patients with routine nursing and responsibility nursing intervention. In terms of adverse emotions, the responsibility nursing group scored lower in SAS and SDS scores than the routine nursing group. Objectively speaking, the medical expenses of hemodialysis are relatively expensive, and the treatment process is long, which brings a burden to the family economy of hemodialysis patients [23]. On the contrary, the whole treatment process will also cause psychological pressure on the patients, which is prone to induce anxiety and depression in patients, resulting in decreased treatment compliance. Responsibility nursing will intervene in the patient's psychology, which, to a certain extent, relieves the patient's resistance to hemodialysis treatment. Besides, the establishment of an optimistic medical attitude helps patients cooperate with the medical staff for treatment and consolidates the therapeutic effect of hemodialysis. After nursing, serum IL-6, hs-CRP, and TNF-*α* of patients in both groups decreased and were even lower in the responsibility nursing group than the routine nursing group. Patients undergoing hemodialysis for a long time may suffer from malnutrition such as inflammation, hypoproteinemia, and muscle protein consumption, which in turn leads to low immunity, aggravating inflammatory reaction, and adversely affecting the prognosis of patients [24, 25]. Through responsibility nursing, the patients' body indexes can be improved as soon as possible to lay a solid foundation for later rehabilitation. In addition, EG was superior to CG in sleep quality and life quality and nursing satisfaction. Routine hemodialysis care only focuses on treating patients' diseases but ignores the feelings of hemodialysis patients. Hence, the effect of nursing treatment is not very significant. Responsibility nursing, on the contrary, also attaches importance to patients' psychological and physiological status. Physical fitness can improve the therapeutic effect, and similarly, the psychological state is directly related to treatment efficacy. Responsibility nursing can help patients establish their determination to overcome diseases and improve their quality of life. When patients receive hemodialysis, the nursing staff provided health education for patients and their families and did a good job of ideological work for their families to gain their understanding and trust, avoid nurse-patient disputes, and ensure smooth treatment. All these measures can validly improve patients' nursing satisfaction with the nursing work provided by the medical staff and finally achieve a significant nursing effect. To sum up, the application of responsibility nursing yields better efficacy in dialysis nursing, which can effectively relieve negative emotions, stabilize the level of inflammation-related indicators in patients, and improve their quality of life, deserving clinical promotion.

## 5. Conclusion

The present study's findings showed that maintaining health, person/client, nursing responsibility, and environment are some of the factors that affect the quality of nursing care in HD departments. The experience of nurses showed that the outcome of the care provided by them was positive for patients. In this study, 120 hemodialysis patients participated and were divided into the control group and experimental group. The two groups were observed and compared for alterations of adverse emotions and inflammatory factors, the incidence of complications, pre-and post-nursing sleep quality, life quality, and patients' satisfaction with nursing. After nursing, the Self-Rating Anxiety/Depression Scale (SAS/DS) scores were lower in the experimental group (EG) than in the control group (CG) (both *P* < 0.05). This proves that, in dialysis care, responsibility nursing for dialysis patients can realistically reduce patients' negative emotions, improve their quality of life, and ensure high-quality dialysis, which is feasible for wide popularization and application in the clinic.

## Figures and Tables

**Figure 1:** Levels of inflammatory factors in two groups of patients. (a) IL-6 levels in two groups of patients; (b) hs-CRP levels in two groups of patients; (c) TNF-*α* levels in two groups of patients; ^*∗∗∗*^*P* < 0.05.

**Table 1:** General information.

	Control group (*n* = 54)	The experimental group (*n* = 66)	*χ* ^2^/*t*	*P*
Gender (*n* (%))			0.1806	0.6709
Male	29 (53.7)	38 (57.6)		
Female	25 (46.3)	28 (42.4)		
Age (years old)	41.92 ± 5.67	43.24 ± 6.04	1.2241	0.2233
BMI (kg/m^2^)	22.52 ± 2.03	22.45 ± 2.17	0.1809	0.8567
Average dialysis time (years)	3.43 ± 0.84	3.58 ± 0.97	0.8945	0.3728
Pathogeny			0.7778	0.8548
Chronic nephritis	21	29		
Hypertensive nephropathy	10	12		
Diabetic nephropathy	15	14		
Polycystic kidney	8	11		
Edema index			0.4104	0.8145
Normal	15	19		
Slight edema	25	27		
Edema	14	20		
Sleep status			0.0219	0.8822
Normal	23	29		
Disorder	31	37		

**Table 2:** Negative emotion scores in two groups.

	SAS score		SDS score	
	Before nursing	After nursing	Before nursing	After nursing
Control group (*n* = 54)	56.51 ± 3.58	42.48 ± 3.14	55.71 ± 4.12	40.58 ± 3.69
Experimental group (*n* = 66)	56.77 ± 3.71	36.14 ± 2.87	55.83 ± 4.36	34.19 ± 2.97
*χ* ^2^/*t*	0.3879	11.5392	0.1537	10.5120
*P*	0.6987	<0.0001	0.8781	<0.0001

**Table 3:** Comparison of sleep quality between two groups.

	Subjective sleep quality		Sleep latency	
	Before nursing	After nursing	Before nursing	After nursing
Control group (*n* = 54)	2.45 ± 0.19	1.52 ± 0.09	2.67 ± 0.26	1.73 ± 0.18
Experimental group (*n* = 66)	2.48 ± 0.12	1.07 ± 0.07	2.58 ± 0.31	1.11 ± 0.09
*χ* ^2^/*t*	0.9183	30.8100	1.6428	24.5000
*P*	0.3603	<0.0001	0.1031	<0.0001

	Sleep duration		Habitual sleep efficiency	
	Before nursing	After nursing	Before nursing	After nursing
Control group (*n* = 54)	2.78 ± 0.64	1.76 ± 0.31	2.59 ± 0.27	1.44 ± 0.31
Experimental group (*n* = 66)	2.75 ± 0.60	1.28 ± 0.24	2.57 ± 0.32	1.06 ± 0.23
*χ* ^2^/*t*	0.2644	9.5590	0.3650	7.7020
*P*	0.7919	<0.0001	0.7157	<0.0001

	Sleep disturbances		Use of sleeping medication	
	Before nursing	After nursing	Before nursing	After nursing
Control group (*n* = 54)	1.92 ± 0.74	1.41 ± 0.55	2.57 ± 0.25	1.27 ± 0.16
Experimental group (*n* = 66)	1.97 ± 0.51	1.12 ± 0.37	2.52 ± 0.19	1.03 ± 0.07
*χ* ^2^/*t*	0.4367	3.4380	1.2442	10.9800
*P*	0.6631	0.0008	0.2159	<0.0001

*P* < 0.05. Likewise, the subjective sleep quality and sleep latency before and after nursing for the EG were 2.48 ± 0.12, 2.58 ± 0.31 and 1.07 ± 0.07, and 1.11 ± 0.09. respectively.

**Table 4:** Quality of life scores of patients in two groups.

	Physical functioning		Material life	
	Before nursing	After nursing	Before nursing	After nursing
Control group (*n* = 54)	58.86 ± 4.25	60.48 ± 3.87	57.25 ± 5.81	61.68 ± 5.22
Experimental group (*n* = 66)	59.24 ± 4.77	68.74 ± 3.54	57.48 ± 5.64	69.43 ± 5.38
*χ* ^2^/*t*	0.4557	12.1930	0.2192	7.9559
*P*	0.6493	<0.0001	0.8268	<0.0001

	Psychological function		Social functioning	
	Before nursing	After nursing	Before nursing	After nursing
Control group (*n* = 54)	56.89 ± 3.26	59.61 ± 3.08	53.87 ± 3.57	58.89 ± 4.14
Experimental group (*n* = 66)	57.06 ± 3.31	64.87 ± 2.97	54.14 ± 3.72	66.71 ± 4.23
*χ* ^2^/*t*	0.2818	9.4923	0.4027	10.1716
*P*	0.7786	<0.0001	0.6878	<0.0001

**Table 5:** Incidence of complications in two groups.

	Dialysis membrane rupture	Mild coagulation	Hypotension during dialysis	Total incidence
Control group (*n* = 54)	4 (7.4)	3 (5.5)	4 (7.4)	11 (20.3)
Experimental group (*n* = 66)	2 (3.0)	1 (1.5)	2 (3.0)	5 (7.5)
*χ* ^2^/*t*				4.2071
*P*				0.0402

**Table 6:** Nursing satisfaction of patients in two groups.

	Environmental satisfaction	Service attitude satisfaction	Technical satisfaction	Lifecare satisfaction	Health education satisfaction
Control group (*n* = 54)	41 (75.9)	38 (70.4)	43 (79.6)	36 (66.7)	39 (72.2)
Experimental group (*n* = 66)	60 (90.9)	63 (95.4)	62 (93.9)	61 (92.4)	60 (90.9)
*χ* ^2^/*t*	5.0031	14.0210	5.5601	12.7210	7.1841
*P*	0.0253	0.0002	0.0184	0.0004	0.0074

## Data Availability

The simulation experiment data used to support the findings of this study are available from the corresponding author upon request.
